# Propranolol Participates in the Treatment of Infantile Hemangioma by Inhibiting HUVECs Proliferation, Migration, Invasion, and Tube Formation

**DOI:** 10.1155/2021/6636891

**Published:** 2021-01-27

**Authors:** Weili Yuan, Xukai Wang

**Affiliations:** ^1^Department of Stomatology, The Fourth Affiliated Hospital of China Medical University, Shenyang, Liaoning, China; ^2^Department of Oral and Maxillofacial Surgery, School of Stomatology, China Medical University, Shenyang, China

## Abstract

**Objective:**

Infantile hemangiomas (IHs) are the most common benign tumors in infancy. The purpose of this study was to study the effects of propranolol on the function of human umbilical vein endothelial cells (HUVECs), in order to preliminarily elucidate the mechanism of propranolol in the treatment of IHs.

**Methods:**

HUVECs were treated with different concentrations of propranolol (30 *μ*M, 60 *μ*M, 90 *μ*M, and 120 *μ*M) with or without VEGF. Their proliferation, migration, invasion, adhesion, and tube formation ability were tested by using CCK-8, wound healing assay, transwell, cell adhesion assay, and tube formation assay. The expressions of HUVECs angiogenesis signaling molecules pERK/ERK, pAKT/AKT, p-mTOR/mTOR, and pFAK/FAK were detected by Western blot.

**Results:**

Compared with the control group, propranolol could significantly inhibit the proliferation, migration, invasion, adhesion, and tube formation of HUVECs. Further studies showed that it could not only inhibit the migration, invasion, and tube formation ability of HUVECs after VEGF induction but also inhibit the phosphorylated protein expressions of angiogenesis-related signaling molecules like AKT, mTOR, ERK, and FAK in HUVECs, with a concentration-dependent inhibitory effect.

**Conclusion:**

Propranolol can inhibit the proliferation, migration, invasion, adhesion, and tube formation of hemangioma endothelial cells; block VEGF-mediated angiogenesis signaling pathway; suppress the expressions of downstream angiogenesis-related signaling molecules; and ultimately achieve the effect of treatment of IHs.

## 1. Introduction

Infantile hemangiomas (IHs) are the most common benign tumors in infants [1]. They grow relatively rapidly during the period from birth to 1 year, and gradually most hemangiomas begin to regress spontaneously after 1 year old, but the entire regression process does not stop until the age of 7 to 10 years. Although IHs are characterized by spontaneous regression, some of them develop so fast that they may cause complications such as infection, ulcers, necrosis, hemorrhage, secondary malformations, and dysfunction [2]. In particular, some refractory hemangiomas in vital parts, such as the airways, joints, face, nipple, fingers, and vulva, do harms to physical and psychological growth. Moreover, a few of complex and severe hemangiomas in crucial parts of the body can cause hemodynamic abnormalities or heart failure and even can be life-threatening [3, 4]. Therefore, for fast-growing IHs with local or systemic complications, researchers prefer to perform corresponding intervention treatment in the early stage to facilitate the spontaneous regression process and to control the growth of hemangiomas and their invasion of surrounding tissues [5]. Although there are massive treatment methods for hemangiomas, all of them have certain adverse reactions [6]. As a result, the treatment of hemangiomas has been a heated topic in clinical and research.

Since 2008, studies have shown that oral propranolol can effectively treat complex and severe IHs [7]. There have been many reports at home and abroad on the successful treatment of IHs by propranolol [8–10], and its efficacy has been confirmed by a large number of clinical observations. Propranolol, a nonselective *β*-adrenergic receptor antagonist, has been reported to be a possibly first-line drug for the treatment of some hemangiomas from accidental discovery. However, there has been not a universally accepted view on the mechanism of propranolol in the treatment of IHs so far. Therefore, it is necessary to have a further study on its mechanism in the treatment of IHs.

According to the literature [11, 12], it could be speculated that the therapeutic mechanism of propranolol in the treatment of hemangioma may be related to the relevant signaling pathways which block angiogenesis, and one of the most important signaling pathways closely related to hemangiomas is the VEGF signal transduction pathway [13]. It was reported in the literature that VEGF bound to its receptor VEGFR and then triggered a series of disorders of intracellular signal transduction pathways such as PI3K/AKT [14], Ras/MAPK [15], NOS [16], PKC [17], and FAK/Paxillin [18], resulting in vascular endothelial cell proliferation, cell survival, cell migration, cytoskeletal rearrangement, vascular penetration, and other processes. In addition, it was said that the expressions of phosphorylated ERK [19], AKT [20], mTOR [21], and FAK [22] were significantly higher in proliferative hemangioma than that in regressive period and normal skin tissues. These researches show that the above signaling molecules are involved in the proliferation of hemangioma, which may be the main activation signal of hemangioma proliferation.

The most typical pathological feature of IHs in clinical practice is the massive proliferation of endothelial cells in tumors. Immortalized human umbilical vein endothelial cells (HUVECs) are characterized by strong proliferation, and the vascular structure in IHs has many similarities with the normal human umbilical vein vascular structure [8–10]. Therefore, in the present study, we selected HUVECs as seed cells for disease model construction to examine the effects of different concentrations of propranolol on ERK/AKT/mTOR/FAK of VEGF-induced angiogenic signaling pathway in HUVECs, hoping to preliminarily clarify the molecular biological mechanism of propranolol in the treatment of IHs and to provide valuable clues and enlightenment for clinical treatment of IHs.

## 2. Materials and Methods

### 2.1. Cell Culture and Treatment

HUVECs were purchased from Shanghai BioHermes Bio&Medical Technology Co., Ltd. (Shanghai, China). Cells were cultured in DMEM complete medium (Gibco, USA) containing 10% fetal bovine serum (FBS, Hyclone, USA) and 1% penicillin/streptomycin (Gibco, USA) and, then, were put into an incubator with 5% CO_2_ at 37°C.

### 2.2. CCK-8 Assay

HUVECs were inoculated in a 96-well cell culture plate with 5000 cells/well. After 24-hour culture in an incubator with 5% of CO2 at 37°C, propranolol serum-free DMEM medium of 30 *μ*M, 60 *μ*M, 90 *μ*M, and 120 *μ*M were added, while 200 *μ*l serum-free DMEM medium was added in the normal control group. The cells were cultured for 24 and 48 hours and then were added with CCK-8 (Keygen Biotechnology Corp., Nanjing, China). Finally, the optical density value (OD value) was measured by 450 nm wavelength microplate reader (BioTek, USA).

### 2.3. Wound Healing Assay

HUVECs were inoculated into 6-well plates, and the cell scratches were made by using 200 *μ*l of pipette tip. After the cell surface was washed twice by adding serum-free medium to remove cell debris, the medium with corresponding concentrations of propranolol (30 *μ*M, 60 *μ*M, 90 *μ*M, 120 *μ*M, and 200 *μ*M) and VEGF (20 ng/mL) was added for further culture for 12 h. Photographs were taken under a 200 × mirror, and the migration distance was measured by using Image-Pro Plus 6.1 software (Media Cybernetics, USA).

### 2.4. Transwell Invasion Assay

Transwell inserts coated with matrigel (Becton, Dickinson and Company, USA) were placed into 24-well plates. 600 *μ*l of complete medium containing 1% of FBS and 20 ng/mL of VEGF were added to the lower chamber, while 400 *μ*l of treated cells from each group was added to the upper chamber (5 × 10^4^ cells/well), cultured on a condition with the temperature of 37°C, 5% CO_2_, and saturated humidity for 24 h. Then, the transwell inserts were removed and rinsed gently with PBS, and those noninvaded cells on the surface of the microporous membrane were wiped off with a cotton swab. Paraformaldehyde was fixed for 20mins at room temperature and stained with 0.1% crystal violet for 3mins. Cells migrating into the lower layer of the microporous membrane were counted under an inverted microscope (200x). Five fields were randomly selected from each sample to count the number of cells.

### 2.5. Cell Adhesion Assay

The cell adhesion assay kit (ScienCell, USA) was used to test the effect of propranolol on cell adhesion ability. Under aseptic conditions, the 48-well plates coated with fibronectin were preheated to room temperature, where 5 × 10^4^/well cells were inoculated and cultured at 37°C for 2 h. At the end of the culture, 200 *μ*l of fresh 0.1% glutaraldehyde was added to each well after they were rinsed with PBS and was fixed at room temperature for 10 mins. Next, 200 *μ*l staining solution was added to each well after which was rinsed with PBS and incubated at room temperature for 30mins on a shaker. Finally, the value of OD595 was measured with a microplate reader.

### 2.6. Tube Formation Assay

Matrigel was added to 96-well plates at 50 *μ*l/well and incubated at 37°C for 30 mins. HUVECs were inoculated into 96-well plates at 10^4^/well, added with various concentrations of propranolol cell adhesion and incubated at 37°C for 8 h. Under an Olympus IX70 inverted microscope, the formation of capillary-like structures was observed, whose extent was quantified by the Image-Pro Plus software.

### 2.7. Western Blot

Total proteins from each group were extracted by the use of NP-40 lysis solution (Beyotime, China). The concentration of the proteins was subsequently determined with the BCA Protein Assay Kit (Beyotime). After being electrophoretically separated by 15% SDS-PAGE, the total proteins transferred to PVDF membranes (Millipore, USA). Then, TBST buffer with 5% nonfat dry milk blocked them for 1 h. Primary antibodies p-FAK antibody (sc-11765, Santa Cruz, USA), FAK antibody (sc-557, Santa Cruz), p-mTOR antibody (sc-101738, Santa Cruz), mTOR antibody (sc-8319, Santa Cruz), p-AKT antibody (sc-135651, Santa Cruz), AKT antibody (sc-8312, Santa Cruz), p-ERK antibody (sc-7383, Santa Cruz), and ERK antibody (sc-135900, Santa Cruz) were added overnight at a dilution of 1 : 400 at 4°C. In comparison, a secondary antibody labeled with horseradish peroxidase (HRP) was used and incubated for 45 mins at 37°C. Color was developed with ECL luminescent solution (Millipore, USA), and after exposure, the results were analyzed by a gel imaging system. Gray scale analysis of protein bands was performed by ImageJ with *β*-actin as an internal protein.

### 2.8. Statistical Analysis

All data were statistically analyzed by the SPSS 22.0 software, and the measurement data were expressed as mean ± standard deviation (SD). One-way ANOVA was used for comparison among multiple groups, while independent sample *T*-test was used for comparison between the two groups. *P* < 0.05 indicated that the difference was statistically significant.

## 3. Results

### 3.1. Propranolol Inhibits HUVECs Proliferation

Compared with the normal control group (NC), 60 *μ*M, 90 *μ*M, and 120 *μ*M propranolol could significantly inhibit the proliferation of HUVECs after treatment for 24 h and 48 h, respectively, with the inhibition rate markedly increasing (Figures 1(a) and 1(b)). The results showed that the higher the concentration of propranolol, the stronger inhibition of HUVECs proliferation is.

### 3.2. Propranolol Inhibits HUVECs Migration

The effects of propranolol on migration and invasion of HUVECs were determined by wound healing assay and Transwell invasion assay. The results in Figures 2(a) and 2(c) showed that compared with the NC group, the migration ability of HUVECs gradually decreased with the increase of propranolol concentration, especially in the 120 and 200 *μ*M propranolol groups for the high concentration. As the proliferation of hemangioma is accompanied by the high expression of VEGF and bFGF [23], VEGF was used to induce HUVECs to simulate the model of hemangioma in vitro. After adding VEGF for 12 h, the migration ability of HUVECs was apparently enhanced. The results in Figures 2(b) and 2(c) showed that propranolol still obviously inhibited the migration ability of HUVECs induced by VEGF after 12-hour culture (*P* < 0.05) in a dose-dependent manner.

### 3.3. Propranolol Inhibits HUVECs Invasion

Transwell assay was performed to detect the effect of propranolol on the invasion ability of HUVECs after VEGF induction. When HUVECs were treated with propranolol for 24 h, the invasion ability of HUVECs decreased significantly with the increasing concentration (30, 60, 90, 120, 200 *μ*M) (*P* < 0.01) (Figures 3(a) and 3(b)).

### 3.4. Propranolol Inhibits HUVECs Adhesion

The results of Figure 4 showed that HUVECs adhesion ability was markedly attenuated with the increasing propranolol concentration (30, 60, 90, 120, and 200 *μ*M) compared with the NC group (*P* < 0.05).

HUVECs were treated with different concentrations (30, 60, 90, 120, and 200 *μ*M) of propranolol, and their adhesion ability was detected by cell adhesion assay. ^∗∗^*P* < 0.01 vs. NC group.

### 3.5. Propranolol Inhibits Tube Formation of VEGF-Induced HUVECs

Furthermore, the ability of propranolol on HUVECs tube formation was tested by angiogenesis assay. In contrast with the NC group, propranolol greatly inhibited HUVECs tube formation in a dose-dependent manner (Figures 5(a) and 5(c)). It was further found that VEGF could distinctly induce HUVECs tube formation. However, with the increasing concentration of propranolol, the tube formation ability of HUVECs and VEGF-induced HUVECs gradually weakened (Figures 5(b) and 5(c)).

### 3.6. Propranolol Inhibits the Activation of VEGF-Induced HUVECs Angiogenesis Signaling Pathways

In order to determine the molecular mechanism of propranolol inhibiting VEGF-induced HUVECs angiogenesis, Western blot was applied to detect the expression of molecules of its signaling pathways in different concentrations of propranolol. The results in Figure 6(a) indicated that propranolol (60, 90, 120, and 200 *μ*M) obviously inhibited that propranolol could notably inhibit the protein expression of p-AKT, p-mTOR, p-ERK, and p-FAK in HUVECs (Figures 6(a) and 6(b)), with a characteristic that the higher propranolol concentration was, the lower protein expression became. All the above results confirmed that propranolol could inhibit the activation of angiogenesis signaling pathways of HUVECs induced by VEGF.

## 4. Discussion

IHs, a common benign tumor in children, are characterized by a complex pathogenesis. Usually not obvious at birth, IHs go through a rapid growth in early infancy [24]. Although they are composed of many different types of cells, it has been speculated in literature that their occurrence and development are mainly brought on by angiogenesis disorders which are caused by abnormal proliferation of vascular endothelial cells [25]. At present, propranolol has been proved to have a good and therapeutic effect on complex and severe IHs. Therefore, it is necessary to make a further research on the mechanism of propranolol in the treatment of IHs, which in turn is helpful to provide valuable clues and enlightenment for clarifying the pathogenesis of hemangioma.

It has been reported that the proliferation, migration, and adhesion of endothelial cells are the key steps of angiogenesis [26]. In our experimental study, we found that propranolol could inhibit the proliferation of HUVECs in a concentration- and time-dependent manner. That meant with the increase of propranolol concentration, their proliferation ability showed a gradually decreasing trend; meanwhile, with the prolongation of propranolol treatment time, the inhibitory effect on the proliferation had a gradually increasing trend. In addition, different concentrations of propranolol could inhibit the migration and invasion of HUVECs in a concentration-dependent manner. It has been confirmed that VEGF is a powerful angiogenesis factor in the occurrence and development process of IHs [27, 28]. As a result, we simulated VEGF induction effect on HUVECs angiogenesis in vitro. It showed that the migration and invasion ability of VEGF-induced HUVECs gradually weakened with the increase of propranolol concentration, and especially in those groups with high propranolol concentration of 120, 200 *μ*M, the migration and invasion ability significantly weakened. It has been said that the invasion and adhesion of tumor cells play an important role in tumor angiogenesis [29]. The results from our experiment also discovered that propranolol at different concentrations could inhibit the adhesion of HUVECs in vitro in a concentration-dependent manner. These results confirmed that propranolol could inhibit angiogenesis by inhibiting the proliferation, migration, invasion, and adhesion of HUVECs.

HUVECs have certain tube formation ability, which is considered as an important reference index for angiogenic function of endothelial cells [30, 31]. As a consequence, this reference index was also included in our experiment to assess the effect of propranolol at different concentrations on the tube formation ability of HUVECs. In this study, the induction of VEGF was able to observably enhance their tube formation ability. Nonetheless, different concentrations of propranolol showed a concentration-dependent inhibitory effect on the tube formation ability of HUVECs without or with VEGF-induction. The result illustrated that propranolol inhibits angiogenesis by inhibiting the tube formation ability of HUVECs.

In the study, it was found that propranolol could significantly inhibit protein expression of the angiogenesis-related signaling pathway molecules, namely p-AKT, p-mTOR, p-ERK, and p-FAK. It was reported in the literature that the expression of p-ERK in the proliferative phase of hemangioma is obviously higher than that in the regressive phase [19]. The biological factors involved in the current hemangioma studies could activate ERK or downstream molecules after ERK was activated. The high expression of p-ERK in proliferative phase suggested that the ERK signaling pathway was involved in the proliferation of hemangioma [32]. According to the literature, the expression of PTEN is negatively correlated with that of p-AKT in IHs, indicating the opposite nature of their expression trend in hemangioma tissues [33]. The expression of PTEN was slightly positive in the proliferative phase of hemangioma but strongly positive in regressive phase, vascular malformation, and vascular endothelial cells of normal skin. The expression of p-AKT was higher in endothelial cells of proliferative hemangioma than in regressive hemangioma. This also suggested that in the proliferative phase of hemangioma, the downregulation of PTEN protein expression may lead to its inability to effectively inhibit the abnormal activation of PI3K/Akt pathway so that the tumor cells could escape from apoptosis and proliferate abnormally, which would promote the occurrence and development of hemangioma [20]. Lv Xin et al. found through an experiment that the high mTOR expression in the proliferative phase of hemangioma might lead to the activation and phosphorylation of p70S6K-*α* and thus promote the rapid proliferation of vascular endothelial cells of hemangioma. Nevertheless, in the regression phase, the mTOR expression was reduced due to the effect of some mechanism, which inhibited the phosphorylation of p70S6K-*α*, blocked the cell cycle in the G0/G1 phase, and then accelerated the apoptosis of vascular endothelial cells of hemangioma, with a tendency of spontaneous regression for hemangioma [21]. Additionally, Zhang Jie et al. discovered that the expression of FAK in proliferative hemangioma endothelial cells was significantly higher than that in degenerative ones and in vascular endothelial cells of normal skin tissues. A large number of FAK expression in proliferative hemangioma cells and the endothelial cell hyperproliferation of hemangioma promoted by the increasing expression of Cyclin D1 pushed the occurrence and development of hemangiomas [22]. All the results demonstrated that propranolol could inhibit the development of hemangiomas by inhibiting the activation of FAK/AKT/mTOR/ERK in signaling pathways of VEGF-induced HUVECs.

## 5. Conclusion

In conclusion, we found that propranolol could decrease the proliferation, migration, invasion, adhesion, and tube formation of HUVECs and inhibit the expression signal proteins closely related to angiogenesis. This study revealed the molecular biological mechanism of propranolol in the treatment of IHs and could provide in-depth experimental and theoretical basis for the pathophysiology of them.

## Figures and Tables

**Figure 1:** Propranolol inhibits HUVECs proliferation. HUVECs were treated with different concentrations (30, 60, 90, 120 *μ*M) of propranolol, and their proliferation ability (a) and proliferation inhibition rate (b) were detected by CCK8. NC: normal control group. ^∗∗^*P* < 0.01 vs. NC group (24 h); ^#^*P* < 0.05 and ^##^*P* < 0.01 vs. NC group (48 h).

**Figure 2:** Propranolol inhibits HUVECs migration. By wound healing assay, the mobility of different concentrations (30, 60, 90, and 120 *μ*M) of propranolol on HUVECs (a) and VEGF-induced HUVECs (b) was measured. (c) Quantitative mobility analysis. Magnification, 200x; ^∗∗^*P* < 0.01 vs. NC group; ^##^*P* < 0.01 vs. VEGF group.

**Figure 3:** Propranolol inhibits of HUVECs invasion. After HUVECs were treated with different concentrations (30, 60, 90, 120, and 200 *μ*M) of propranolol for 24 h, cell invasion ability was measured by Transwell (a). (b) Quantitative analysis of invasive cell counts. Magnification, 200x; ^∗∗^*P* < 0.01 vs. VEGF group.

**Figure 4:** Propranolol inhibits of HUVECs adhesion.

**Figure 5:** Propranolol inhibits tube formation of VEGF-induced HUVECs. Angiogenesis assay was performed to detect the tube formation ability of HUVECs (a) and VEGF-induced HUVECs (b) after 8-hour treatment with different concentrations (30, 60, 90, 120, and 200 *μ*M) of propranolol. (c) Quantitative analysis of the number of HUVECs tube formation. Magnification, 200x; ^∗∗^*P* < 0.01 vs. NC group; ^##^*P* < 0.01 vs. VEGF group.

**Figure 6:** Propranolol inhibits the activation of VEGF-induced HUVECs angiogenesis signaling pathways. After VEGF-induced HUVECs were treated with different concentrations of propranolol (30, 60, 90, 120, 200 *μ*M), (a) the expression of p-AKT/AKT, p-mTOR/mTOR, p-Erk/Erk, and p-FAK/FAK was detected by Western blot. (b) Gray analysis of protein bands. ^∗^*P* < 0.05 and ^∗∗^*P* < 0.01 vs. VEGF group.

## Data Availability

Some or all data, models, or code generated or used during the study are available from the corresponding author by request.
